# Construction of Digital Teaching Resources of British and American Literature Using Few-Shot Learning and Cloud Computing

**DOI:** 10.1155/2022/4526128

**Published:** 2022-06-26

**Authors:** Hui Zhang, Fang Zuo

**Affiliations:** ^1^School of Foreign Languages, Sichuan Technology and Business University, Meishan 620000, China; ^2^Foreign Language School of Chengdu University of Traditional Chinese Medicine, Chengdu 611137, China

## Abstract

British and American literature is a compulsory course for English majors in Chinese colleges and universities. It plays an important role in cultivating students' aesthetic consciousness and moral cultivation, improving students' humanistic quality and cultural taste, and shaping students' complete personalities. With the rapid development of cloud technology and mobile Internet technology, mobile learning based on mobile devices will become an important direction of mobile Internet technology applications. Based on cloud computing, this paper studies the construction of digital teaching resources of the British and American literature. Through the experiment on the learning simplicity of literature courses for English majors, it is found that during the learning period of 40 people, the average proportion of the most difficult is 16.3%, the average proportion of the second difficult is 35.2%, and the average proportion of the easier is 18.5%. Compared with the next difficulty, the proportion of difficulty is the highest, followed by the easy and finally the most difficult. As one of the core technologies of cloud computing, data split storage technology adopts measures such as isomorphism and interchangeability of computing nodes, redundant storage, and multicopy fault tolerance to ensure the high security and reliability of user data and users do not have to worry about data loss and virus invasion. As a new generation of technical means, cloud computing can realize the unified management and scheduling of distributed and heterogeneous resources and provide a new development direction for promoting the coconstruction and sharing of the British and American literature digital teaching platforms in higher vocational colleges and truly realizing national learning and lifelong learning.

## 1. Introduction

British and American literature, as a required course for Chinese English majors in their third year, serves a critical function in broadening students' cultural horizons and cultivating high quality. It is critical in developing students' aesthetic consciousness and moral development, as well as strengthening their humanistic quality and cultural taste and forming their entire personality [1, 2]. The authorized curriculum of the postgraduate entrance test for English majors includes British and American literature. In recent years, this course's information has been included in the CET8 test content [3]. There are a variety of causes for the marginalization of British and American literature at colleges and universities, but there are two major reasons. It is a result of the contemporary mercantilist social climate. Some colleges and universities continue to add practical and effective Applied English courses such as business English, economic and trade English, financial English, legal English, and computer English when teachers are strictly prohibited in order to reduce the number of class hours of English and American literature courses as much as possible [4, 5]. Students dig deeper into and investigate the contents of literary works, fully integrating the collected information into their English knowledge system. They enhance their English level in addition to enhancing their literary literacy [6].

Mobile learning based on mobile devices will become an important path for mobile Internet technology applications with the rapid growth of cloud technology and mobile Internet technology. Based on the cloud platform, the mobile digital resource platform mines related learning needs and habits using cloud computing technology's storage space and data analysis capabilities [7, 8], allowing students and teachers to access the network resource cloud service platform and obtain resources at any time and from any location. The process of data processing is relocated from personal computers or servers to computer clusters on the Internet, which is dubbed “cloud” [9], using the high-speed transmission capabilities of cloud computing on the Internet. Cloud computing has accelerated the evolution of information technology and IT application mode, fundamentally altered working and business modes in the traditional mode, and increased resource utilization and computing speed, simplifying software, business processes, and access services. Cloud computing provides computation, services, software, and other services to a large number of users at the same time, and maintaining data security is the foundation for gaining consumers' trust. Data sharing storage technology, as one of the core technologies of cloud computing, employs features [10, 11] such as isomorphic and interchangeable computing nodes, redundant storage, multicopy fault tolerance, and other features to ensure that user data are secure and reliable, and users do not have to worry about data loss or virus intrusion [12, 13]. The core objective of cloud computing is to share the processing and storage resources of each node in the cloud, to deliver to end-users, and to take the required computer resources as its main role. Cloud computing will inevitably find its way into more and more digital teaching tools for British and American literature [14, 15]. In the cloud computing mode, by building a common cloud platform for digital teaching resources of British and American literature, the links within schools, between schools, and between schools and enterprises can be closer, and educational information resources can be effectively integrated and shared. With this platform, schools and enterprises can also effectively save human and material resources, realize resource complementarity, and promote two-way cooperation. As a new generation of technical means, cloud computing can realize the unified management and scheduling of distributed and heterogeneous resources so as to provide a new development direction for promoting the coconstruction and sharing of British and American literature digital teaching platforms in higher vocational colleges and truly realizing national learning and lifelong learning.

This article studies and innovates the above problems from the following aspects:

1. A cloud server model of English and American literature digital teaching resources based on cloud computing is proposed. The digital teaching resource base based on cloud computing also reduces the difficulty of operation, and users can easily use the resource base without mastering complicated software operations. Digital resources store information in data centers to meet the needs of students and teachers; memory management is used to organize and manage data from cloud service end to mobile client application end; the management layer realizes the interaction between security control and memory management through the cloud management platform.
2. A digital teaching resource construction system of British and American literature based on cloud computing is constructed. Through the digital teaching resources construction system of British and American literature, a resource information database and a resource catalogue database are established to manage resources and provide support for the rapid retrieval of resources. Because resources need to be shared with different databases, it is necessary to establish common technical standards and build database platforms according to the same specifications to prevent data incompatibility.

The article is divided into five parts, and the organizational structure is as follows: Section 1 introduces the research background and present situation of digital teaching resources of British and American literature and puts forward and summarizes the main tasks of this paper.  Section 2 introduces the related work of digital teaching resources of British and American literature at home and abroad.  Section 3 introduces the algorithms and models of cloud computing.  Section 4 introduces the realization of the digital teaching resources of British and American literature and compares the performance of the system through experiments.  Section 5 is the full-text summary.

## 2. Related Work

### 2.1. Research Status at Home and Abroad

Zhang L et al. put forward that there are many problems in the teaching materials of British and American literature. First, most of the teaching materials are of single style and not readable, which is difficult to attract students' interest; second, the replacement speed of teaching materials is too slow. Many teaching materials are old in content and viewpoint, which can not meet the students' desire to know the latest things; third, the textbook pays too much attention to the indoctrination of knowledge and lacks enlightenment, ignoring the cultivation of students' intelligence and ability [16]. Li proposed that the purpose of literature course is to cultivate students' ability to read, appreciate, and understand the original works of English literature, master the basic knowledge and methods of literary criticism, improve students' basic language skills and humanistic quality through reading and analyzing British and American literary works, and enhance students' understanding of western literature and culture [17]. Yi proposed that the construction of a digital teaching platform of British and American literature can integrate the existing human resources and academic resources, use the huge text, video, and audio information to increase students' knowledge, cultivate students' correct learning methods, and improve learning efficiency. In turn, it can enable students to join the classroom teaching links and the construction of a digital teaching platform, highlight their subjectivity and exercise their reading ability, scientific research ability, and expression ability [18]. Shan proposed that in view of the problems existing in the current British and American literature course, I think it is necessary to make use of the current rich network resources and use modern teaching methods to improve the teaching effect of the British and American literature course, so as to play its due role in higher education and get rid of its marginalization [19]. Ma and Bo proposed to improve students' basic language skills and humanistic quality and enhance students' understanding of western literature and culture by reading and analyzing British and American literary works [20]. Campbell put forward that it is necessary for teachers to optimize and reform the existing teaching mode of British and American literature, make full use of modern educational technology and network multimedia, update teaching contents, improve teaching efficiency, and cultivate students to master effective learning methods [21]. Al-Zoube et al. pointed out that some teachers of English and American literature courses started to use multimedia in the teaching process, but many of them just showed the contents of textbooks in the form of courseware. This kind of “textbook moving” courseware did not give full play to the advantages of multimedia, so it was not attractive [22]. Hwang and Li put forward the compiling characteristics of foreign English and American literature textbooks, analyzed the shortcomings in domestic textbooks, and put forward corresponding reform suggestions [23]. Yang pointed out that the contents of most English and American literature textbooks are relatively outdated, but the use of network resources can make up for this deficiency. Teachers can collect, download, and sort out some resources to meet students' needs from the Internet and selectively integrate the latest contents and research results of British and American literature into the lecture notes in time [24]. Li pointed out that literary appreciation ability, cross-cultural ability, and critical thinking ability are essential basic abilities for foreign language majors. Whether students have these abilities depends largely on the quality of teaching materials used in literature courses and the teaching effect on teachers and students [25].

### 2.2. Research Status of Digital Teaching Resources of the British and American Literature Based on Cloud Computing

This article analyzes the construction of digital teaching resources of British and American literature under cloud computing, the opportunities, and challenges faced by British and American literature teaching in Chinese universities and discusses how to reform the teaching mode and improve the teaching efficiency under cloud computing. Building and sharing a British and American literature teaching resource library using cloud computing technology is critical for China's talent development so that high-quality educational resources may be popularized and more students can benefit from them. It is difficult for pupils to understand abstract concepts solely through linguistic interpretation during the educational process. Cloud computing technology can help concretize abstract ideas and simplify complex situations, allowing you to achieve twice the outcome with half the effort. The use of cloud computing technology, on the other hand, offers teachers with a new digital teaching resource teaching system of British and American literature, which encourages teachers to challenge traditional teaching notions and promote constant innovation in all parts of education. Improving their English language skills is also conducive to creating a literary learning atmosphere integrating knowledge and interest, stimulating their interest in learning, and cultivating their autonomous learning habits. Therefore, the teaching of British and American literature can fully reflect its humanistic knowledge and improve its teaching quality.

## 3. Algorithm and Model of Cloud Computing

Cloud computing is a network made up of a large number of computers that can offer consumers the necessary computer services. This supercomputing mode reflects the future development trend of computer applications and is the newest development achievement of distributed computing, parallel computing, and grid computing in the field of computer science. “Computing” refers to a “computing resource pool” in cloud computing, while “cloud” refers to multiple networks that provide resource services. Cloud computing service providers are in charge of virtualized device management and operation, as well as dynamic resource deployment, real-time scheduling, and autonomous recycling, among other things. Virtualization technology is used to make cloud computing a reality. In general, the computer element runs on a real basis, but in virtualization technology, the computing element runs on a virtual basis. Cloud computing resources are always developing dynamically, and different computer terminals can add different types of information to the cloud for other users to download and share. End consumers do not need to understand how the cloud works, let alone have expert knowledge, and everything is as simple as connecting to the Internet.

Cloud services can govern and administer a vast number of educational information resources with the use of cloud computing. Any learner requires only a cloud-connected computer or a mobile terminal device that operates on a 3G or WiFi network. In any place and at any time, they can get the learning resources and services he needs from the cloud resource library in real time. They can also use cloud resources to debate a specific problem with teachers and specialists, making virtual network learning a reality. The operating difficulties are also reduced by the digital instructional resource library based on cloud computing. The resource library is simple to use and does not need users to grasp sophisticated software processes. The user interface is welcoming, and the experience is very humanized, which can help to boost the learning effect significantly. The following are the basic components of the mobile digital cloud server: The data center's information is stored in digital resources, which are used to suit the demands of students and teachers. From the cloud service to the mobile consumer application, memory management is used to organize and manage data. Through the cloud management platform, the management processing layer accomplishes the connection between security control and memory management. The cloud server model of digital teaching resources of British and American literature is shown in Figure 1.

Allocate virtual machines to each application according to the resource vector *R*=(*R*_1_,…, *R*_*j*_,…, *R*_*c*_) allocated to each application output by the application monitoring program module so as to minimize the total allocation cost. In other words, the purpose of this module is to assign the virtual machine of each application that minimizes the objective function as follows:

(1) $$\begin{array}{c} C=\min\left(\sum_{i=1}^{m}\cos\;t\cdot N_{i}\right), \end{array}$$

where *m* is the number of applications, cos  *t* is the operation cost vector of virtual machines, each item corresponds to the allocation cost of each type of virtual machine, *N*_*i*_ is the virtual machine vector allocated to application *i* and *N*_*i*_=(*n*_*i*1_,…, *n*_*ij*_,…, *n*_*ic*_), *n*_*ij*_ is the number of *j*-type virtual machines allocated to application *i*, and cos  *t* · *N*_*i*_ represents the cost of allocating virtual machine vector *N*_*i*_ to application *i*.

According to the assumption in this article, the number of each type of virtual machines in the data center is limited; that is, there is an upper threshold. The threshold vector of each type of virtual machine is defined as *N*^max^=(*n*_1_^max^,…, *n*_*j*_^max^,…, *n*_*c*_^max^) and has the following relationship:

(2) $$\begin{array}{c} \sum_{i=1}^{m}n_{ij}\leq N_{j}^{\max},\;1\leq j\leq c. \end{array}$$

The number of resources allocated to each application should meet the resource requirements determined by the application monitoring module, namely,

(3) $$\begin{array}{c} \sum_{j=1}^{c}n_{ij}\cdot V_{j}^{CPU}\geq R_{i}^{CPU},\;1\leq i\leq m,\\ \sum_{j=1}^{c}n_{ij}\cdot V_{j}^{\text{memory}}\geq R_{i}^{\text{menory}},\;1\leq i\leq m,\\ \sum_{j=1}^{c}n_{ij}\cdot V_{j}^{\text{network}}\geq R_{i}^{\text{network}},\;1\leq i\leq m. \end{array}$$

At the same time, the total resources of all virtual machines deployed on physical machines cannot exceed the total resources of all physical machines, so there is the following relationship:

(4) $$\begin{array}{c} \sum_{i=1}^{m}\sum_{j=1}^{c}n_{ij}\cdot V_{j}^{CPU}\leq \sum_{j=1}^{n}p_{j}^{CPU},\\ \sum_{i=1}^{m}\sum_{j=1}^{c}n_{ij}\cdot V_{j}^{\text{memory}}\leq \sum_{j=1}^{n}p_{j}^{\text{memory}},\\ \sum_{i=1}^{m}\sum_{j=1}^{c}n_{ij}\cdot V_{j}^{\text{network}}\leq \sum_{j=1}^{n}p_{j}^{\text{network}}. \end{array}$$

By solving the above model with the constraint method, we can get the virtual machine allocation vector with the lowest total cost, and each virtual machine allocation vector corresponds to the virtual machine allocation situation of each application, that is, what kind of virtual machines are allocated and the number of virtual machines allocated.

Therefore, a teaching resource model with the best energy consumption of heterogeneous servers can be established:

(5) $$\begin{array}{c} \text{minimize}\sum_{i\in P}\left(H_{i}\cdot E_{i}^{\text{dynamic}}+E_{i}^{\text{static}}\right), \end{array}$$

where *E*_*i*_ is the energy consumption of physical server *p*_*i*_. It can be concluded that the constraints on energy consumption are

(6) $$\begin{array}{c} E_{i}^{\text{static}}+H_{i}\cdot E_{i}^{\text{dynamic}}\leq E_{i}^{\text{Max}}\left(1\leq i\leq n\right). \end{array}$$

Among them, *E*_*i*_^Max^ is the maximum energy consumption that physical server *p*_*i*_ can bear; that is, the actual energy consumption of the physical server *p*_*i*_ must be less than or equal to *E*_*i*_^Max^.

Cloud computing provides resources, services, and platforms for users. It can provide users with safe, convenient, and efficient services as needed at any time, anywhere, and anyway. It has the characteristics of superscale, safety and reliability, on-demand service, and strong versatility. Cloud computing is a service-centered networked computing resource sharing pool. The main body of its architecture includes the application layer, platform layer, infrastructure layer, and virtualization layer, which provide software as a service, platform as a service, and infrastructure as a service, respectively. On-demand access through service support. In addition, the client and management together constitute the architecture of cloud computing. The architecture of cloud computing is shown in Figure 2.

The architecture of cloud computing is mainly divided into six layers:

① Application layer
  In the application layer, services are provided through software applications, which interact with the client through web service and other technologies to realize the corresponding functions.
② Platform layer
  Based on the virtualization layer, the platform layer plays an important role in connecting the preceding and the following. It is responsible for responding to the requests sent by the application layer, using distributed technology to process massive data in parallel, dynamically allocating various resources of the virtualization layer according to the requests, and providing platform services is a key step to improving efficiency.
③ Virtualization layer
  The virtualization layer is based on the infrastructure layer, which virtualizes the resources provided by the infrastructure layer. It can also be understood as the “multitenant” of the infrastructure layer, which makes efficient and rational use of the resources provided by the infrastructure according to the processing needs sent by the platform layer.
④ Infrastructure layer
  The infrastructure layer provides the necessary resources for the virtualization layer, including software resources, network resources, and hardware resources. This layer can expand and optimize management based on the database.
⑤ Client
  The client is used for human-computer interaction, including user interface and machine interface.
⑥ Management
  The management manages the as a service at all levels. Through good user management technology, users can quickly log in under safe conditions and facilitate the unified management of accounts by administrators. Resource management is the overall allocation of all resources.

Cloud computing is to centralize computers in different parts of the country and realize collaborative work through the network. Users can get the services they need only through the network. In this way, there is no need to add a lot of computer hardware equipment and install various software programs for certain needs, which directly saves a lot of costs. Cloud computing users will have their own resource requirements. In order to make the resources requested by users run, it is necessary to allocate the specific resources requested by users to them. Typical cloud computing resource provision strategies include the strategy based on lease theory and dynamic multilevel resource pool, the strategy based on economics college, the strategy based on general optimization algorithm, and the optimal strategy based on random integer programming.

## 4. The Construction and Realization of Digital Teaching Resources of the British and American Literature

### 4.1. Teaching Resource Construction System under Cloud Computing

After the learner is authenticated and authorized, the cloud platform analyzes the learning contents of the digital teaching resources of British and American literature according to the learner's historical track and displays them in a list, thanks to the cloud platform's data analysis and processing capability. It may learn at any time and from any location, which is incredibly handy for students and teachers and boosts their efficiency. Many large network companies have now developed a number of relevant processes and standards to ensure customer data security, provided various solutions for schools based on their needs, built a cloud platform that meets the needs of schools, and created a private “public resource cloud” for schools to better serve their teachers and students. You may also specify multiple levels of permissions to link with external units to create a “hybrid cloud” that allows you to share resources. The operating system and computer hardware are targeted for virtualization in the instructional resource creation system platform. Application virtualization includes simulation, simulation, and interpretation technology. Resource virtualization focuses on specific system resources such as network resources, storage, and memory; resource virtualization focuses on specific system resources such as network resources, storage, and memory. Virtualization technology optimizes resource use and eliminates resource waste. Both software and hardware are capable of performing well. Computers solve real problems at a far faster rate. Light resources, accessible resource deployment, diversified resource channels, ubiquitous resource acquisition, and speedy resource browsing should be characteristics of the cloud-based digital teaching resources development system for British and American literature. On the basis of knowledge deconstruction, lightweight development of teaching resources is carried out to fulfill the needs of fragmented learning, MOOC teaching, and flipped classroom. The particle size of resources not only follows the instructional principles but also helps with network transmission. We should take full advantage of the resource pool's openness and boost its interactivity when building a cloud-based system of digital teaching tools for British and American literature. Despite the fact that the cloud stores a wide range of educational and teaching resources, users may quickly access them and set up storage, editing, calling, querying, and downloading. It is the primary driving factor behind the English and American literature digital teaching resource creation system. The construction will lack scale if the application scope is too narrow; the promotion will be worthless if the application is ineffective.

The building and application of digital teaching resources must be led by the construction and improvement of British and American literary resources, which should begin with the construction and improvement of British and American literature resources and formulate a professional curriculum system based on the professional talent training plan, which includes professional core courses, professional support courses, and expansion courses. Professional core courses are those that reflect professional core competencies, while professional support courses are those that provide support and basic support to the core courses. The efficient management of digital teaching resources in the resource cloud for British and American literature plays a critical role in increasing user experience and promotion effect. Rapid resource retrieval, fair resource scheduling, resource approved access, and so on are all aspects of management. The resource information database and resource directory database are established through the digital teaching resource construction system of British and American literature to manage resources and give support for speedy resource retrieval. Because separate databases must share resources, consistent technological standards must be established and a database platform built to the same specifications to avoid data incompatibility. Because the digital teaching resource construction system based on cloud computing for British and American literature is still in its early stages of development and research, the technology is not fully mature, and various standards are not fully unified. It is critical to establish corresponding technical specifications.

### 4.2. Experimental Results and Analysis

In this experiment, the students' interest and liking for digital teaching resource databases were investigated, and the interest and liking of secondary vocational school students for digital teaching resource database were basically the same. The degree of students' interest in the resource pool is shown in Table 1. The degree of students' liking for the resource pool is shown in Table 2.

From Tables 1to 2, it can be seen that 58.8% and 55.2% of students are very interested in and like the resource bank, 28.3% and 30.7% are interested and like, 7.8% and 9.3% are generally interested and like, and 4.7% and 4.6% are not interested and dislike, respectively. In terms of content construction, we should comply with the characteristics and teaching methods of secondary vocational schools, update the content in time, and keep pace with teaching, and students can find the content they want in time to truly serve teachers' teaching and students' learning. The resource bank is mainly for teaching. In the design and construction, we should widely solicit the opinions of students and teachers, especially the direct and in-depth participation of front-line teachers. In addition to the systematic design of the content in line with the characteristics of secondary vocational teaching, it also needs to be designed in terms of management to facilitate teachers' teaching management and teacher-student interaction on the resource database platform.

In this experiment, the first three aspects of students' simplicity in learning English and American literature courses are analyzed. Two experiments were conducted to compare the most difficult and the second most difficult, respectively, and the total time spent by students studying the course after class was compared. The experimental results are shown in Figures 3 and 4.

From Figures 3to 4, it can be seen that the three learning points of traditional language, cultural background, and text content have different difficult relationships in students' activities of learning English and American literature. According to the experiment of English major students' ease of learning literature courses, it is found that during the period of 40 students, the average proportion of the most difficult is 16.3%, the average proportion of the next difficult is 35.2%, and the average proportion of the easier is 18.5%. Compared with the next difficult one, the proportion of the difficulty in learning is the highest, followed by the easier one, and finally the most difficult one. Most students have greater difficulties than language barriers in understanding the content of literary works and related knowledge reflected by them. Only a small number of students' language barriers exceed the cognitive barriers of text content and related knowledge.

In this experiment, during the classroom teaching, after the teacher has finished explaining the works preliminarily, the students are divided into several groups, each with 4–6 people, to discuss a certain problem in the preview tips, respectively. According to the order in which these teaching AIDS appear in the teaching process, the order is as follows: (1) discuss in groups; (2) scenario demonstration; (3) simulation teaching. Group discussion aims to improve the efficiency of preview before class by training students' ability to collect effective information and communicate. Once again, we conducted three experiments to compare English majors' preferences for the response teaching mode. The experimental results are shown in Figures 5, 6, and 7.

As can be seen from Figures 5to 7, for each single teaching auxiliary means of group discussion, scenario demonstration, and simulated teaching, when the number of students is 50, the average satisfaction rates of group discussion, scenario demonstration, and simulated teaching are 34.6%, 34.9%, and 37.6%, respectively. The results of this experiment reflect that the students affirmed the three teaching aids adopted under the guidance of reception response theory. The improvement of students' learning quality and learning interest shows the effectiveness of the above auxiliary teaching means: that is, to strengthen students' understanding of literary texts and promote the exchange and communication between learning subjects so as to obtain a better literary teaching effect.

## 5. Conclusions

It is of great significance for China's talent training to build and share the British and American literature teaching resource library through cloud computing technology so that high-quality educational resources can be popularized and more students can enjoy high-quality educational resources. The development and utilization of digital teaching resources of British and American literature based on cloud computing is not only conducive to creating a multimode humanistic teaching environment in which multiple meaningful symbols work together, enhancing the intuition and vividness of teaching, mobilizing students' multiple senses to participate in language information perception, and effectively improving English language skills but also conducive to creating a literary learning atmosphere in which knowledge and interest are combined and stimulating students' interest in learning, Cultivate students' autonomous learning habits, improve literary literacy, fully realize the teaching objectives of British and American literature, and reflect the teaching knowledge of British and American literature. Through the experiment on the difficulty and ease of learning literature courses for English majors, it is found that among the 40 students, the average proportion of the most difficult is 16.3%, the average proportion of the second difficult is 35.2%, and the average proportion of the easier is 18.5%. Compared with the next difficulty, the proportion of learning difficulty is the highest, followed by the easier, and finally the most difficult. Various materials provided by the cloud computing British and American literature teaching platform improve students' literary appreciation ability and critical judgment ability, enhance students' scientific research ability, expression ability, and innovation ability and improve students' comprehensive quality.

## Figures and Tables

**Figure 1:** Cloud service model of British and American literature digital teaching resources.

**Figure 2:** Architecture of cloud computing.

**Figure 3:** Learning effects of public English courses at different levels of difficulty.

**Figure 4:** Learning effects of professional English courses at different levels of difficulty.

**Figure 5:** English majors' satisfaction with the reception response teaching model on 10% training samples.

**Figure 6:** English majors' satisfaction with the reception response teaching model on 20% training samples.

**Figure 7:** English majors' satisfaction with the reception response teaching model on 30% training samples.

**Table 1:** Questionnaire on students' interest in the resource database.

Degree	Very interested	Be interested	Commonly	Uninterested
Number of people	425	204	56	34
Proportion	58.8%	28.3%	7.8%	4.7%

**Table 2:** Questionnaire on students' preference for resource database.

Degree	Like it very much	Like	Commonly	Dislike
Number of people	397	222	67	33
Proportion	55.2%	30.7%	9.3%	4.6%

## Data Availability

The data used to support the findings of this study are available from the corresponding author upon request.
